RETRACTED

# Focal Microscopy Observe the Mechanism of Gegen Qinlian Decoction Treating Type 2 Diabetic Nephropathy in Nude Mice

**DOI:** 10.1155/2022/1636301

**Published:** 2022-08-08

**Authors:** Fei Zheng, Juan Xu, Hao Gu

**Affiliations:** ^1^Department of Pharmacy, Medical Supplies Center of PLA General Hospital, the Second Military Medical University of PLA, Beijing 100853, China; ^2^Department of Pharmacy, Medical Supplies Center of PLA General Hospital, Shenyang Pharmaceutical University, Beijing 100853, China; ^3^First People's Hospital of Chenzhou City, Southern Medical University, Chenzhou, 423000 Hunan, China

## Abstract

The incidence of diabetes is increasing year by year; among them, the rising trend of T2D is particularly obvious, and because it has many complications and poor prognosis, it has become one of the diseases that seriously endanger human health. Gegen Qinlian Decoction (GQD) has achieved good results in the treatment of type 2 diabetes (T2D). It can not only improve the anti-insulin effect of nude mice with type 2 diabetic, but also has the characteristics of small side effects and remarkable curative effect; it can improve the function of tissues and organs by multiple target spots and multiple ways. The method was to raise 30 nude mice with high fat and high sugar and inject small doses of streptozotocin (STZ). The treated nude mice were randomly divided into rosiglitazone group, Gegen Qinlian group, and model group, normally rearing 10 nude mice as a control group. The model group and the blank group were treated with 0.9% sodium chloride solution at 10 mL/kg, and the rosiglitazone group was intragastric administration with 3 mg/kg rosiglitazone solution. The GQD group was treated with 18.2 g/kg GQD, once a day, and lasting for 4 weeks. Use blood glucose meter to detect the FBG content in nude mice, use the radioimmunoassay to detect the amount of FINS, and calculate HOMA-IR. Use immunoenzyme linked assay method to detect the level of serum inflammatory factors. The experimental results showed that compared with the model group, the FBG of the rosiglitazone group mice was significantly decreased; the levels of the rosiglitazone group and the Gegen Qinlian group were significantly lower. Therefore, it is concluded that GQD can treat T2D in nude mice.

## 1. Introduction

Diabetes (diabetes mellitus) is one of the most common endocrine diseases; clinical diabetes is divided into many types, which are the most common T2D and diabetes T2D; in particular, in recent years, all over the world in a rapid increase, if not timely treatment of patients, the deterioration will cause serious damage to the patient's body organs [1]. Chinese herbal medicines usually contain large amounts of chemicals that can be converted into more complex metabolites in the body, but for many years, traditional detection methods have been able to detect only a few dozen metabolites. With the advancement of science and technology, scientists have used high performance liquid chromatography (HPLC) and Fourier transform ion cyclotron resonance mass spectrometry (UHPLC-FT-ICR-MS) methods to analyze rat plasma, urine, and feces. 174 compounds were detected in the metabolites, of which 107 compounds were prototypes and 67 compounds were metabolites. At the same time, metabolic pathways in rats were also found, including hydrogenation and hydrolysis [2, 3].

RETRACTED

Pueraria scutellariae, traditional Chinese medicine prescriptions for CD and clinical use, have achieved good hypoglycemic effects in the treatment of T2D. Gegen scutellariae syrup (GGQLT-CS) can promote the therapeutic effect of HepG2 cells in the pathogenesis process. Insulin has positive effects on glucose consumption, reducing PEPCK activity, increasing hepatic glycogen content, regulating HepG2 cell glucose metabolism, and improving hepatic insulin resistance [4]. Network pharmacology also revealed that the effective mechanism of Gegen Qinlian Decoction in the treatment of T2D was mostly related to anti-inflammatory and antioxidant stress [5]. The study on the model of obese rats with spontaneous T2D also showed that Gegen Qinlian Decoction can improve insulin resistance and regulate inflammatory cells. Therefore, cytokines are related to the treatment of T2D by Gegen Qinlian Decoction. Therefore, in this paper, the type 2 diabetes model was replicated by feeding a high-fat and high-sugar diet and a small dose of streptozotocin, and the effect of Pueraria Scutellariae on insulin resistance and inflammatory factors in type 2 diabetes model rats was investigated, aiming to regulate inflammatory cytokines through Pueraria lobata and Scutellaria baicalensis, improve T2D insulin resistance, and lay a more profound theoretical basis for future CD treatment.

Qi Wang studied the intestinal permeability of 42 active components of Gegen Qinlian Decoction by LC/MS/MS and found the highest content of alkaloids in Rhizoma coptidis [6]. Qiao Xue studied the metabolic pathways of single Chinese herbal components in Gegen Qinlian Decoction by extracting the compounds in the formula and summarized a set of practical methods for identifying the metabolites of Gegen Qinlian Decoction [7]. Ling Xiao used miniature pigs as a model, used E. coli to cause diarrhea in miniature pigs, and tested pig feces to determine the content of 9 main components and CD in Pueraria Scutellariae [8]. Zhong Wen used Pueraria Scutellariae and CD to study the influence of traditional Chinese medicine raw materials and production processes on the consistency of traditional quality [9]. In order to study Pueraria Scutellariae and its main active components and CDon rat liver microsomal isoenzyme activities, Liu Zihua used in vitro liver microsome culture technology and the analysis method of probe substrate metabolites to monitor the linear relationship formed between rat body protein concentration, incubation time, and metabolite amount [10]. The data of these studies are not comprehensive, and the results of the studies are still open to question, so they cannot be recognized by the public and thus cannot be popularized and applied.

RETRACTED

## 2. Proposed Method

### 2.1. Confocal Laser Scanning Microscope

Confocal laser scanning microscope (CLSM) uses laser as the scanning light source to quickly scan and image point by point, line by line and side by side. If the tissue sample contains a substance that can excite fluorescence, it will directly return to the spectrometer of the original incident light path through the opposite direction after the excitation fluorescence is exposed and focus through the detection pinhole, and the focused light is PMT [11].

### 2.2. T2D

T2D (formerly known as non-insulin-dependent diabetes) is a serious and difficult disease that has long plagued Americans, affecting about 8 percent of American adults. Due to the drastic changes in Chinese people's lifestyle and the increasing incidence of diabetes, T2D is gradually becoming a high incidence in Chinese people. Its treatment can prevent some devastating complications, but usually cannot restore normal blood glucose or eliminate all the adverse consequences [12]. Through cell culture and mouse model experiments, scientists have found that obesity causes endoplasmic reticulum stress. This stress inhibits insulin receptor signaling through hyperactivated kinase (JNK), manifesting at the ER stress molecule, cellular, and organismal levels, and is central to peripheral insulin resistance and T2D drug-controlled features.

Gegen Qinlian Decoction is often used in the treatment of T2D and has achieved a good effect in lowering blood sugar. Experimental studies have also proved that it can improve the insulin resistance of T2D rats. The study of spontaneous T2D model in obese rats revealed that the mechanism of action of Scutellaria baicalensis and CD in the treatment of T2D is related to anti-inflammatory and antioxidative stress. It has the effect of improving Pueraria Scutellariae and CD insulin resistance and regulating inflammation. Therefore, cytokines are related to Gegen Huangqin combined with Huanglian Decoction in the treatment of T2D, which can effectively relieve insulin resistance in patients, promote human insulin secretion, and also effectively improve clinical symptoms [13].

RETRACTED

According to traditional Chinese medicine, T2D can be understood as “quenching thirst”, characterized by excessive drinking, eating and urination [14]. Modern medicine regards T2D as a metabolic disease characterized by hyperglycemia, which is caused by defective insulin secretion or insulin dysfunction. Metabolic disorders are mainly caused by congenital or acquired enzyme defects, mainly due to cardiovascular disease, kidney disease, or excessive nucleic acid decomposition. The clinical manifestations are excessive or low blood uric acid, gout, and neurological symptoms. Relevant studies have shown that serum uric acid level is positively correlated with chronic complications in patients with T2D. Uric acid is an independent risk factor for atherosclerotic lesions, which can accelerate the development and progress of renal lesions in patients with T2D. If the level of uric acid in human body is too high, if it is not controlled in time, it will interfere with the function of insulin, lead to insulin resistance, and then lead to the increase of blood glucose. Therefore, the development of T2D has nothing to do with the disorder of sputum metabolism.

## 3. Experiments

### 3.1. The Experimental Materials

40 SPF nude mice were selected as animal subjects in the experiment. The humidity in the breeding environment was kept at 50% ~ 60%, the room temperature was kept at 22~ 26°C, and the light time was adjusted according to the normal circadian rhythm.

Drug GQD, composed of radix puerariae, scutellaria, baked liquorice root, and Coptis chinensis, was prepared as decoction and heated in water bath at 37 °C before use.

The main reagents are streptozotocin (STZ), purchased by Sigma Company, and insulin radioimmunoassay kit, purchased by Beijing Huaying Biological Co., Ltd. Tnf-alpha, il-6, il-1 beta, and McP-1 ELISA Kit were purchased by R&D corporation (USA). The blood glucose meter was purchased from Yuyue Medical Equipment Co., Ltd. (Shanghai); the Fresco cryogenic centrifuge was purchased from Thermo (USA); the MultiSkan3 microplate reader was purchased from Thermo (USA); the micropipette was purchased from Eppendorf (Germany).

One hundred patients with diabetes were selected as the subjects of this study, and one hundred patients were randomly divided into the control group (metformin) and the experimental group (Gegen Qinlian Decoction), with 50 patients in both groups.

Control group is composed of the following: 24 males and 26 females, aged between 39 and 64 years, with an average age of50.35 ± 1.69 years and an average course of disease of6.52 ± 2.71 years.

RETRACTED

Experimental group is composed of the following: 26 males and 24 females were aged between 38 and 65, with an average age of49.65 ± 2.71 years and an average course of disease of6.29 ± 2.91 years.

### 3.2. The Experimental Method

After 40 nude mice were fed for 1 week, they were randomly divided into two groups: 10 mice were used as blank group, 30 mice were used as model group, the blank group was fed with ordinary diet, and the model group was fed with high-fat and high-sugar diet. After continuous feeding for one month, nude mice in both groups were injected with STZ solution configured with sodium citrate buffer with a pH of 4.4 at a dose of 30 mg/kg (note: make sure the nude mice are in an empty state). After one week, blood was collected from the tail vein of the nude mice (ensure that only water was given to the nude mice within 12 hours prior to blood collection without feeding), and fasting blood glucose of the nude mice was measured by glucometer. If the blood glucose content ranged from 16.7 mmol/L to 30 mmol/L, the model was considered successful. The successfully modeled nude mice were randomly divided into three groups, with 10 nude mice in each group, respectively, labeled as the model group control group, Gegen Qinlian decoction group, and rosiglitazone group.

On the second day of the drug treatment group, nude mice in four groups were given the following dosage by gavage: In the blank group, 0.9% sodium chloride solution was 10 mL/kg; model group, 0.9% sodium chloride solution 10 mL/kg; Gegen Qinlian Decoction group, 18.2 g/kg; and rosiglitazone group, 3 mg/kg.

After the end of specimen collection and treatment, make sure that only the nude mice are fed with water and no feed within 12 hours before blood collection, quickly collect blood from the tail of all the nude mice, and measure fasting blood glucose with a glucometer. After the nude mice were anesthetized, they were treated with drugs, and then blood was taken from the abdominal aorta of the nude mice, left standing for half an hour, and rotated at a high speed of 3,500 revolutions per minute after the blood was taken. Centrifuge in a high-speed centrifuge for 15 minutes to separate the serum, transfer the supernatant to an EP tube and label it, and store it in a -20°C refrigerator for future testing.

The serum insulin content in the four groups of nude mice was detected by radioimmunoassay in accordance with the operating instructions attached to the kit. 100 microliters of serum and standard substances were taken from four groups of nude mice and labeled. 100 microliters of antibody and 100 microliters of 125i-ins were added to each tube, thoroughly mixed, and placed in a water bath at 37 °C for two hours. Add 500 microliters of immune separator to each tube, fully mix, centrifuge at 3,500 RPM for 15 minutes, remove the supernatant, detect the CPM value of precipitation, and calculate the level of FINS for each group of rats. Calculate the insulin resistance index: HOMA − IR = (FBG × FINS)/22.5.

RETRACTED

Step 1. Add 5 micron total RNA and 1 micron Oligo (dT) (10 microns) into 0.2 ml centrifuge tube

Step 2. Place the above mixture in the PCR instrument, adjust the temperature to 65 °C, heat it for 10 minutes, take it out, and put it on ice immediately, and cool it for 2~3 minutes

Step 3. Under ice bath conditions, add 5× m-mulv reaction buffer (8 mu/Ll), d NTP mixture(5 mu/L), m-mulv reverse transcriptase (1 mu/L), and DEPC water (20 mu/L) to the centrifugal tube

Step 4. Centrifuge briefly to let the reactant sink to the bottom of the tube, and place it in 37 °C for one-and-a-half hours to synthesize the first chain of cDNA, and then heat it at 65 °C for 5 minutes to terminate the reaction.

The treatment method for the control group was as follows: taking metformin from HebeiTiancheng Pharmaceutical Co., Ltd. (National Drug Approval No.: H13021647), orally, 500 mg each time, twice a day.

Treatment in the experimental group: On the basis of the control group, Gegen Qinlian decoction was used for treatment. GQD basic medicine soup contains six grams of processed licorice, six grams of coptis, thirty grams of Pueraria root, and twenty grams of Scutellariae. For patients with deficiency of Qi and Yin, additional pollen, American ginseng, Poria cocos, and Atractylodes are added into the formula. For patients with desiccated lung and stomach heat, the formula is added with Anemarrhena, Poria cocos, raw land, Cortex Phellodendri, and other herbs. For patients with stasis and stagnation and dampness-heat interaction, alisma, ligusticum chuanxiong, coix seed, and salvia miltiorrhiza were added into the formula. For patients with damp-heat type, Poria cocos, Shengdi, black ginseng, and Ophiopogon japonicus were added to the internal prescription. All the ingredients in the recipe were boiled into pharmaceutical juice, and patients in both groups were treated with one course of treatment, one course of treatment for two months, one dose per day (keep 200 ml), one dose per time, one dose in the morning, and one dose in the evening.

## 4. Result and Discussion

### 4.1. Analysis of the Diseased Population of T2D and the Use of Different Drugs

The purpose of research on the incidence of T2D patients is to understand that the current need for treatment of the disease is very large. One hundred patients with diabetes were selected as the subjects of this study, and one hundred patients were randomly divided into the control group (metformin) and the experimental group (Gegen Qinlian decoction), with 50 patients in both groups. The control group consisted of 24 males and 26 females, aged between 39 and 64 years, with an average age of 50.35 ± 1.69 years and an average course of disease of 6.52 ± 2.71 years. The experimental group included 26 males and 24 females, aged between 38 and 65 years, with an average age of 49.65 ± 2.71 years and an average course of disease of 6.29 ± 2.91 years. After fasting for one night, participants received an oral glucose tolerance test and measured fasting and 2-hour blood glucose levels. Previously, diagnosed diabetes was determined on a self-reported basis. Among people aged 20 to 39, 40 to 59, and over 60, the prevalence of diabetes increased with age (3.2%, 31.5%, and 40.4%, respectively), as shown in Table 1 and Figure 1. The prevalence of diabetes in urban and rural residents (11.4%) was higher than that in rural residents (8.2%). The incidence of diabetes mostly occurs in the elderly group (over 40 years old).

RETRACTED

The changes were obtained by observing various indexes of nude mice by focusing microscope.  Table 2 and Figure 2 are the naked comparative results of murine FBG, FINS, and HOMA-IR. From the data in Table 2 and Figure 2, it can be seen that the FBG, FINS, and HOMA-IR of the model group are significantly higher than those of the blank group. Fasting blood glucose is referred to as FPG, which refers to the blood collected before breakfast after an overnight fast (at least 8-10 hours without any food, except for drinking water), and the blood glucose value detected is the most commonly used test index for diabetes, which reflects pancreatic islet B cells. After 4 weeks of continuous administration, compared with the model group, the FINS content and HOMA-IR in the Puerarin Qinlian decoction group decreased significantly (*P* < 0.05), suggesting that Puerarin Qinlian decoction can improve the insulin resistance of T2D, mainly by improving the sensitivity of insulin. Compared with the model group, the FBG in the Gegen Qinlian decoction group decreased (20.58 vs. 24.26), but there was no significant difference.

### 4.2. Experimental Results of Gegen Qilian Decoction

1. Healthy SD male nude mice were divided into normal control group, T2D model group, and Gegen Qinlian decoction treatment group. In addition to the normal group, all nude mice were fed with high-fat streptozotocin to establish the animal model of T2D. The model was established after three weeks of continuous lavage, and urine samples were extracted 12 hours after the last lavage. HPLC/MS-IT-TOF method was used to determine and describe the differences in urine metabolism between each group. Network pharmacology, systematic pharmacology, and metabolomics have consistently shown that Gegen Qinlian decoction can treat T2D with multiple targets and multiple pathways. Especially in recent years, Pueraria Scutellariae and CD have played an important role in the treatment of intestinal inflammation and can significantly inhibit the production of various inflammatory cytokines. Compared with the model group, the CD serum levels of 1-6 L and L-1b in the Pueraria Scutellaria group were significantly decreased. The results showed that Pueraria Scutellariae and CD could improve the level of serum inflammatory factors in nude mice in type 2 diabetic rats and play a role in insulin resistance. Comparison of serum inflammatory factors in nude mice in each group is shown in Table 3 and Figure 3
2. When Gegen Qinlian decoction was used in the treatment of nude mice with T2D, the level of some endogenous small molecule metabolites at the metabolomics level returned to normal, and the level of disease characteristics and indicators was significantly improved, achieving a better therapeutic effect on the whole. The set of physical and chemical indicators to compare is shown in Table 4 and Figure 4

RETRACTED

## 5. Conclusions

The treatment of diabetes is inseparable from the contribution of Gegen Qinlian Decoction and focusing microscope. Through comprehensive experimental tests, it can be seen that Gegen Qinlian Decoction has an obvious effect on the treatment of T2D. The content of FBG in nude mice was detected by blood glucose meter, the amount of FINS was detected by radioimmunoassay, and HOMA-IR was calculated. The results showed that the FBG of the rosiglitazone group was significantly lower than that of the model group (*P* < 0.01). Therefore, it is concluded that the effect of Gegen Qinlian Decoction on T2D in nude mice may be related to the inhibition of the release of inflammatory factors; after Gegen Qinlian Decoction treats T2D nude mice, some endogenous small molecule metabolites are recovered at the metabolomics level normal, disease characteristics and index levels were significantly improved, and overall good therapeutic effect was achieved; by dividing healthy SD male nude mice into normal control group, T2D model group, and Gegen Qinlian Decoction treatment group, it was inferred that the occurrence of T2D and purine metabolism were inferred. Closely related, nucleotides are the key targets. Through the multi-targets of Pueraria Scutellariae and CD to regulate abnormal purine metabolism, it can even cause systemic disease disorder and restore it to normal levels. The amount of data in this study is small, so the results of the study may have some chance.

RETRACTED

## Figures and Tables

**Figure 1:** Rates of diabetes in different age groups.

**Figure 2:** FBG, FINS, and HOMA-IR in nude mice of each group were compared.

**Figure 3:** Comparison of serum inflammatory factors in nude mice in each group

**Figure 4:** Set of physical and chemical indicators to compare.

**Table 1:** Rates of diabetes in different age groups.

Age	20~39	40~59	>60
Probability of illness (%)	3.2	31.5	40.4

**Table 2:** FBG, FINS and HOMA-IR in nude mice of each group were compared.

Group	FBG (mmol/L)	FINS (mIUl/L)	HOMA-IR
Control group	5.12 ± 0.53	14.89 ± 3.83	3.45 ± 0.78
Model group	24.26 ± 5.02	21.09 ± 2.36	23.09 ± 5.33
Rosiglitazone group	17.36 ± 4.05	17.72 ± 2.06	13.72 ± 5.06
Gegen and Qinlian soup group	20.58 ± 2.83	18.09 ± 2.96	16.09 ± 3.96

**Table 3:** Comparison of serum inflammatory factors in nude mice in each group.

Group	TNF-*α*	IL-6	IL-1*β*	MCP-1
Control group	0.44 ± 0.66	3.89 ± 0.53	60.45 ± 8.78	130.45 ± 12.78
Model group	2.26 ± 1.02	9.09 ± 1.36	123.09 ± 25.33	173.09 ± 25.33
Rosiglitazone group	0.96 ± 0.25	5.72 ± 1.36	89.72 ± 10.06	149.72 ± 12.06
Gegen and Qinlian soup group	1.58 ± 0.43	7.09 ± 1.46	93.09 ± 14.96	158.09 ± 10.96

**Table 4:** Set of physical and chemical indicators to compare.

Group	FPG (mmol /L)	Scr (mmol /L)	BUN (mmol /L)	TG (mmol /L)
Control group				
Before the treatment	9.44 ± 2.52	93.52 ± 19.84	8.16 ± 1.28	3.03 ± 0.26
After the treatment	6.21 ± 1.58	66.35 ± 11.53	5.13 ± 1.15	1.27 ± 0.17
Experimental group				
Before the treatment	9.42 ± 2.61	95.48 ± 18.89	8.23 ± 1.31	3.10 ± 0.17
After the treatment	7.23 ± 2.21	81.62 ± 19.89	6.38 ± 1.18	1.74 ± 0.22

## Data Availability

No data were used to support this study.
